# Robust Detection Model of Vascular Landmarks for Retinal Image Registration: A Two-Stage Convolutional Neural Network

**DOI:** 10.1155/2022/1705338

**Published:** 2022-07-30

**Authors:** Ga Young Kim, Jae Yong Kim, Sang Hyeok Lee, Sung Min Kim

**Affiliations:** ^1^Department of Medical Biotechnology, Dongguk University, 32, Dongguk-ro, Ilsandong-gu, Goyang-si, Gyeonggi-do, Republic of Korea; ^2^Department of Ophthalmology, Dongguk University Ilsan Hospital, 27, Dongguk-ro, Ilsandong-gu, Goyang-si, Gyeonggi-do, Republic of Korea

## Abstract

Registration is useful for image processing in computer vision. It can be applied to retinal images and provide support for ophthalmologists in tracking disease progression and monitoring therapeutic responses. This study proposed a robust detection model of vascular landmarks to improve the performance of retinal image registration. The proposed model consists of a two-stage convolutional neural network, in which one segments the retinal vessels on a pair of images, and the other detects junction points from the vessel segmentation image. Information obtained from the model was utilized for the registration. The keypoints were extracted based on the acquired vascular landmark points, and the orientation features were calculated as descriptors. Then, the reference and sensed images were registered by matching keypoints using a homography matrix and random sample consensus algorithm. The proposed method was evaluated on five databases and seven evaluation metrics to verify both clinical effectiveness and robustness. The results established that the proposed method showed outstanding performance for registration compared with other state-of-the-art methods. In particular, the high and significantly improved registration results were identified on FIRE database with area under the curve (AUC) of 0.988, 0.511, and 0.803 in S, P, and A classes. Furthermore, the proposed method worked well on poor quality and multimodal datasets demonstrating an ability to achieve high AUC above 0.8.

## 1. Introduction

Image registration transfers images which are acquired at different times and viewpoints, or by different modality, and represents them in a single coordinate system [1]. It has been widely applied to medical image analysis to obtain useful information from combining several data sources. In particular, retinal image registration is an essential process in diagnosis and treatment of various retinal diseases [2, 3]. Clinically, combined information acquired from several retinal images is valuable for fully understanding about diseases. Registration can provide support for determining correct therapy and increasing treatment success rate by applying it for detecting lesions changes, tracking disease condition, and monitoring therapeutic response.

Manually comparing two images (the reference and sensed images) is a laborious task and takes a significant amount of time. To solve this problem, many researches have proposed computer-aided automatic registration methods, and they have helped to reduce the task time and burden on ophthalmologists. They can be categorized into two types: feature-based and intensity-based methods [4–6].

The feature-based method detects features including region, edge, and line [7]. The correspondence between the features are calculated for image registration. In this method, the features should be distinct and spread over the image region [1]. Also, they should have common characteristics even if images are taken from a different angle or direction, or some other unexpected change occurs. The feature-based method is robust for illumination variations, because features hold information on a high level.

The intensity-based method statistically compares the entire region or subregion of the reference and sensed images. To calculate the similarity and match the image pair, a variety of metrics can be used including cross-correlation, mutual information, phase correlation, sum of absolute values of differences, and entropy correlation [4]. This method is fit for simple transformation problems. However, its performance can suffer from the heavy computational complexity and illumination variations, because these may lead the significant changes in the intensity of images [8].

In the retinal image registration problem, pairs of images to be compared may have large differences in their intensity distribution. Even if the retinal image is obtained from the same person and a similar environment, noise and illumination artifact may occur. Also, the development of lesions such as exudate, microaneurysm, and drusen may induce changes in the image. Overall, the feature-based method is considered more robust than the intensity-based method in these situations, and therefore, we mainly focused on the feature-based method for the registration of the retinal image.

For retinal image registration, various feature-based methods have been proposed to detect keypoint sets in previous studies [9–11], and many have used retinal vessel information such as vasculature trees, bifurcation points, and crossover points which can be acquired by manual or automatic methods. These retinal vessel features are known to be stable and satisfy the characteristics [9] that features should have. Importantly, retinal vessels are spread throughout the entire image region, and they are structurally distinct with dark and low intensity on the retinal image. As well, vessels are a common element even in diverse situations and conditions, because they are relatively invariant to the intensity variance [12]. Therefore, this study selected retinal vessel information for image registration.

This study proposed a robust detection model of vascular landmarks for retinal image registration. The proposed model consists of a two-stage convolutional neural network, with one being for vessel segmentation and the other for junction detection. For registration, the keypoints were designated by using the obtained vascular landmark points, and descriptors were calculated using orientation features based on SIFT algorithm [13]. Then, the keypoints were matched and the image pair was registered. The proposed method was evaluated on five databases and seven evaluation metrics to identify its clinical effectiveness and robustness. The experiment was conducted using TensorFlow frameworks on Intel Core I7-7700 K CPU and GeForce GTX 1080 Ti GPU.

The remainder of this paper is organized as follows: Section 2 introduces prior related studies.  Section 3 presents the proposed method including image preprocessing, vascular landmark detection model, and registration algorithm.  Section 4 presents the datasets and evaluation metrics which were used to perform and evaluate the proposed method, and this section also contains the experimental results. Lastly, Section 5 contains the discussion and conclusion.

## 2. Related Work

A number of earlier studies have proposed diverse registration methods that can be applied to retinal image. In [14], similar vessel structure was used for retinal image registration. Bifurcation and terminal points were detected from the centerline of skeletonized retinal vessels. Then, similar vessel regions on the image pair were matched based on the Hungarian matching algorithm. Ramli et al. [15] proposed a D-saddle detector to extract feature points on retinal vessel with diverse contrast and size. This method could detect features even on low-quality regions by combining the conventional saddle detector with multiresolution difference of Gaussian pyramid. It showed higher success rate and accuracy compared with GDB-ICP, Harris-PIIFD, and H-M. Chen et al. [16] used the angle and length features between bifurcation points and connected branches. These features were normalized to be less affected by the image transformation. They also proposed a shortest path algorithm to obtain clear vascular trees by connecting or removing the isolated ridge on the initial segmented retinal vessel region with width of one pixel. In addition, many other studies [5, 17–19] have actively conducted registration research based on the information provided by junction points such as bifurcation, trifurcation, crossover, and terminal.

Despite these efforts, several studies showed limitation in registration performance. Retinal image registration methods based on vascular information are heavily dependent on the vessel segmentation performance. However, automatic vessel segmentation is a difficult process because of the poor and inhomogeneous contrast of retinal images. It is extremely challenging to detect junction points using existing filter-based methods. Although many studies have applied the skeletonization algorithm prior to junction detection, a great deal of vascular information may be missed or incorrect junctions can be obtained in this process. Furthermore, it is hard to match the reference and sensed images with only lengths and angles, because there are many similar junction points on the retinal images and these points are often indistinguishable from image to image. To address the limitations of these previous studies, this study proposed a robust detection model of vascular landmarks for retinal image registration.

## 3. Material and Methods

### 3.1. Image Preprocessing

Contrast-limited adaptive histogram equalization (CLAHE) was applied to the original retinal images before they were input to the proposed model. The retinal images were taken in different environments and situations, and as such, they were likely affected by illumination, noise, etc. Because this could negatively influence registration performance, the pixel intensity on the retinal images was equalized by CLAHE with tile size of 8 × 8.

In addition, the images were augmented during the training process of the proposed detection model to prevent the overfitting problem and efficiently train the model. The two types of methods including flip and rotation were used in this study. One flipped the image horizontally or vertically, or both, and the other rotated the image with different angles between 0° and 360°.

### 3.2. Vascular Landmark Detection Model

The goal of this study was to achieve registration of retinal image pairs obtained from the same person. For that, this study detected vascular landmarks based on a deep learning model. The proposed model involves a two-stage deep network, which segments retinal vessels and detects vessel junctions based on the U-net [20] and RetinaNet [21] algorithms. In detecting vessel junction, the initial areas which include junction points were detected, and then, they were calibrated to improve the detection performance.

#### 3.2.1. Vessel Segmentation Network

In the first part of the model, the retinal vessel region on the retinal image was segmented by an individual network named as vessel segmentation network (VSN). This network was designed based on U-net which was proposed by Ronneberger et al. [20]. The architecture of VSN is presented in Figure 1.

The VSN consists of the convolution based downsampling path and the transposed convolution based upsampling path. In the downsampling path, as the levels go deeper, the sizes of the feature maps are reduced by half and higher-dimensional features are obtained. Meanwhile, the size of these feature maps was recovered in the upsampling path. In other words, the downsampling path captured the context of the retinal image to extract advanced features, and the upsampling path was conducted for more precise localization. Additionally, the upsampled feature map was concatenated with the downsampling path to obtain the localization information.

The VSN includes a multi-input module and a connected convolution module. The multi-input module fed image datasets to the fore part of the downsampling path on each level as shown in Figure 2. The preprocessed image was resized and convoluted to match with input data of the correspondence level. Then, it was concatenated with input data of the former level. This module could make the model learn richer context features by providing image information and fusing it with a feature map of each level. The connected convolution module was applied to improve performance by connecting the feature maps in same level (Figure 3). The feature maps were calculated by applying 3 × 3 convolution, batch normalization, and ReLU function, and the input feature map and acquired second feature map were concatenated. This structure enabled the VSN to share information between different steps in the module and train the complex features.

In this study, different hyperparameters of the model were compared, and optimal conditions were set to alleviate the overfitting problem and efficiently train the model. Epoch was 100 and learning rate was 5 × 10^−6^. Adam and cross entropy were applied for the optimizer and loss function.

#### 3.2.2. Junction Detection Network

Junction detection network (JDN) was designed based on the RetinaNet [21] for the detection stage. The JDN was trained to detect vascular junction points consisting of bifurcation and crossover to apply them as keypoints for image registration. As shown in the architecture of the network (Figure 4), the JDN included the downsampling and upsampling paths.

Downsampling consisted of five levels, and it was constructed using the ResNet-50 [22]. Multiple residual layers were involved in the ResNet module on each level, and these layers efficiently extracted the feature maps through a specific process. First, residual function (*R*) was performed to the input value*x*_*i*,*j*_ (*j^th^* layer on *i^th^* level) in order, 1 × 1, 3 × 3, and 1 × 1 convolution. In residual function, the ReLU function was involved between convolution operations. Then, the calculated value (*R*(*x*_*i*,*j*_)) was added to the input value of the layer as shown in Equation (1). Before this process, the dimension of these two values were matched by using identity mapping (*I*). Finally, the *x*_*i*,*j*+1_ was calculated by operating the ReLU function to the added value. This residual layer was repeated on each level. The output feature map on the last residual layer, named *C*_*i*_, was used for further processing. The size of the feature map {*C*_1_, *C*_2_, *C*_3_, *C*_4_, *C*_5_} was reduced by half as the level became deeper.

(1) $$\begin{array}{c} x_{i,j+1}=\text{ReLU}\left(R\left(x_{i,j}\right)+I\left(x_{i,j}\right)\right). \end{array}$$

To minimize the computational load, only three *C*_*i*_(*i* ∈ {3,4,5}) were used in the upsampling process. These *C*_*i*_ values were applied the 1 × 1 convolution and upsampled by a factor of 2 using 3 × 3 transposed convolution. Then, a merged feature map (*M*_*i*_) was obtained by connecting convoluted and upsampled values in the same level with element-wise addition method as shown in Figure 4. This structure compensated for the missing local information.

In the next process, three new feature maps denoted as *P*_*i*_(*i* ∈ {3,4,5}) were generated by applying 3 × 3 convolution to the *M*_*i*_. This convolution was used to reduce the aliasing effect which may occur due to the lost information in the previous process [23], and *P*_6_ and *P*_7_ were obtained by conducting the 3 × 3 convolution to *P*_5_ with stride 2. The spatial size was reduced 0.5 times.

From the acquired feature maps, the anchor boxes with a predefined shape were applied to detect the junction point. The length of base anchors (BA) were set for the feature map (*P*_3_ − *P*_7_). Then, multiple anchor boxes were calculated from each of the base anchors with two scales (*S*) and three aspect ratios (AR), which were, respectively, set as {2^0^, 2^1/2^} and {1, 2, 0.5} in this study. The height and width length of the anchor box were calculated by using Equations (2) and (3). The maximum number of boxes was set at 200, because the number of junction points was less than 200 on retinal images in the empirical study.

(2) $$\begin{array}{c} H_{m,n}=\frac{\text{BA}\times S_{m}}{\sqrt{{\text{AR}}_{n}}}, \end{array}$$

(3) $$\begin{array}{c} W_{m,n}=\text{BA}\times S_{m}\times \sqrt{{\text{AR}}_{n}}, \end{array}$$

where *m* and *n* are the index number of scale and aspect ratio, respectively.

These anchor boxes were classified and regressed in the two subnets (Figure 4). These subnets consist of five sequential 3 × 3 convolutions. The classification subset used the focal loss [21] as loss function, while the smooth *L*1 loss was applied for the regression of the anchor boxes. The JDN was trained by integrating these two loss functions and optimized using momentum with cosine learning rate decay [24].

#### 3.2.3. Calibration

The vascular landmark points for registration were detected with VSN and JDN. For the registration step, the detected points play an important role by matching corresponding points between image pairs. The detection performance could affect the registration performance. Therefore, this study calibrated the vascular landmark points before the registration step. First, the subimage was obtained by cropping the image based on the detected vascular landmark points. Then, the centerline of the vessel was acquired by skeletonizing the vessel region [25], and the points were calibrated by taking into account that three or more branches are met in vascular junction points. For all pixels in the subimage, the neighbor vessel pixel was counted, and the junction points were revised.

### 3.3. Image Registration

The vascular landmark points detected by the above model were used for image registration. For the reference and sensed images, the regions within a distance of five pixels from the junction points were designated as keypoints, and descriptors were calculated using orientation feature based on SIFT algorithm [13]. The similarity between the descriptors for two images was evaluated by using Euclidean distance. Then, keypoints were matched by comparing the distance and finding the closest pair. In this process, some keypoint pairs were ignored if the distance ratio between the nearest distance and second closest distance was higher than a certain threshold. The optimal threshold was chosen as 0.84 through the empirical study.

To register the pair of retinal images, the 3 × 3 homography matrix was calculated from the matched keypoints by considering the rotation, scale, shearing, reflection, translation, and perspective [26]. Outliers which could interrupt the registration were removed by applying random sample consensus algorithm [27]. The acquired matrix transformed the sensed image as described in Equations (4) and (5) to register two images. The coordinate of the transformed pixel (*a*′, *b*′) was calculated from the original pixel (*a*, *b*) of the sensed image.

(4) $$\begin{array}{c} a^{\prime }=\frac{h_{1,1}\times a+h_{1,2}\times b+h_{1,3}}{h_{3,1}\times a+h_{3,2}\times b+1}, \end{array}$$

(5) $$\begin{array}{c} b^{\prime }=\frac{h_{2,1}\times a+h_{2,2}\times b+h_{2,3}}{h_{3,1}\times a+h_{3,2}\times b+1}, \end{array}$$

where *h*_*p*,*q*_ is an element of the homography matrix in row (*p*) and column (*q*).

## 4. Experiments and Results

### 4.1. Dataset

In this study, retinal images were acquired from a total of five public databases to train the proposed model and verify the performance. Details about each database are as follows.

The DRIVE [28] database was used to train and test the VSN and JDN. It contains 40 retinal images which have been divided into train and test datasets with 20 images each. These images were provided in JPEG file format with 768 × 584 resolution. This database also provided the ground truth dataset obtained by manual segmentation task performed by human observers. They were instructed by an ophthalmologist and requested to segment regions as retinal vessels when they were convinced to a degree of certainty of greater than 70%. This ground truth dataset was used to evaluate the segmentation performance of the proposed method.

Although the DRIVE database offered a prominent dataset with regard to vessel segmentation, it did not involve information on vessel junctions. Therefore, the RetinaCheck [29, 30] database was supplementally collected and used for junction detection. This database provided the ground truth of bifurcation and crossover points on the retinal images of the DRIVE database which was annotated by three experts. The RetinaCheck database also provided the ground truth for the IOSTAR database [29, 30] which was obtained by i-Optics B.V. on the Netherlands.

The FIRE [31] database was used for the evaluation of registration performance, because it contains not only pairs of retinal images acquired from the same patients but also the correspondence data relevant for each image pair. The image dataset consists of 134 image pairs acquired from 39 patients, with resolution of 2912 × 2912 pixels. Also, the images were categorized into 3 classes (S, P, and A) according to the characteristics of the image pairs such as approximate overlap, anatomical changes, and registration application.

To verify the robustness of the proposed method, two other databases were applied which were supplied by Köhler et al. [32] and Alipour et al. [33]. The first database contains 18 image pairs which consist of two images of good and poor quality obtained from the same person. The providers mentioned that the images with poor quality were affected by a defocused camera setting. The second database provided 60 fluorescein angiography and retinal images acquired from 30 healthy people and 30 patients with diabetic retinopathy. These databases were applied to confirm two things: whether the proposed method will be affected by image quality and whether it will show reasonable performance even with multimodal images. However, these two databases did not involve the ground truth for registration. Therefore, the correspondence points were manually detected by the authors after training by an ophthalmologist in Dongguk University in the Republic of Korea. The ground truth obtained in this way was double checked by an ophthalmologist for reliability of the dataset.

### 4.2. Performance Evaluation

The performance of the proposed method was evaluated in three parts, and these consisted of vessel segmentation, junction detection, and registration. For each part, different evaluation metrics were used to quantitatively analyze the performance, and the results were compared with other state-of-the-art methods.

Confusion matrix-based evaluation approaches were used for vessel segmentation and junction detection. This is a table which lays out the results of the predicted class from the model and groups each actual label into four elements as shown in Table 1. These elements consist of true positive (TP), true negative (TN), false positive (FP), and false negative (FN), and various performance measurements can be calculated based on these elements. In this study, sensitivity (TP/(TP + FN)), specificity (TN/(TN + FP)), and accuracy ((*TP* + *TN*)/(*TP* + *TN* + *FP* + *FN*)) were used for the VSN, and the JDN was evaluated by precision (TP/(TP + FP)), sensitivity, and F1 score (2TP/(2TP + FP + FN)). The sensitivity and specificity measure how well the network correctly identifies the positive and negative into actual classes, respectively. The sensitivity is also known as recall in the detection problem. The precision calculates the ratio of well-detected regions to all regions predicted as positive. The accuracy is the proportion of TP and TN in the entire elements, and F1 score represents the harmonic mean of precision and sensitivity. Also, the performance of the VSN was evaluated by using the area under the curve (AUC) of the receiver operating characteristic (ROC) curve which was plotted based on the sensitivity and specificity.

For the registration score, measurements proposed by Hernandez-Matas et al. [10] were applied in this study. In this method, the success rate was obtained for the error threshold in the range from 0 to 25. From this, a curve was plotted in which the *x*-axis is the error threshold and *y*-axis is the success rate. The AUC of this curve was used for quantitative evaluation.

### 4.3. Experimental Results for Retinal Vessel Segmentation

The VSN was evaluated on the DRIVE database. The network was trained with 20 images from the database, and another 20 images were used for testing. The obtained results were compared with other state-of-the-art methods using four evaluation metrics consisting of sensitivity, specificity, accuracy, and AUC.  Table 2 lists the retinal vessel segmentation performance of the proposed VSN as well as other unsupervised/supervised methods. The VSN achieved the highest AUC of 0.982 outperforming other diverse methods. For the other metrics, superior performance of the VSN was also demonstrated for sensitivity, specificity, and accuracy with results of 0.805, 0.982, and 0.966, respectively.

### 4.4. Experimental Results for Retinal Vessel Junction Detection

The RetinaCheck database was used to test the JDN. This study calculated the detection results involving precision, sensitivity, and F1 score according to the type of input image as shown in Table 3. The color image is the original RGB image, and the grayscale image refers to the green channel which generally showed distinct retinal tissues among the three channels. The vessel image indicates the manually segmented binary image representing 1 for retinal vessel pixels and 0 for other pixels. The experimental results on the color image had a relatively low F1 score of 0.752, and the grayscale image showed an increased F1 score by about 0.022. The performance was improved to over 0.8 in all three metrics by using the vessel image for input data. The optimal results for precision, sensitivity, and F1 score were 0.809, 0.853, and 0.831, respectively.

Also, the RetinaCheck database was applied to the previously trained VSN and JDN for evaluation of the proposed vascular landmark detection model. This allowed an evaluation of the overall performance of the proposed vascular landmark detection model, including the series of processes from segmenting the retinal vessel on the retinal image to detecting junction points using the acquired vessel image. Then, the results were compared with other methods as shown in Table 4. The results of the COSFIRE were written by citing the contents of [30]. For the BICROS, the results using 2-D Gabor wavelet segmentation method are displayed in Table 4. The method proposed in this study performed better than all four other methods on the DRIVE image dataset for all three metrics. Furthermore, it also demonstrated a significant F1 score of 0.646 on the IOSTAR dataset.

### 4.5. Experimental Results for Retinal Image Registration

The retinal image registration performance of the proposed method was evaluated on the FIRE database. For pairs of images, junction points were extracted using the proposed model. Next, these points were used to register the reference and sensed images.  Figure 5 presents the resulting images of each process for the FIRE image dataset, and Table 5 shows the experimental results of the proposed method and five other methods. The information in the 3^rd^~5^th^ rows of Table 5 were written with reference to the paper of Hernandez-Matas et al. [10]. The proposed method exhibited a superior AUC. Especially, these results were 0.010 and 0.143 higher in S and A classes compared with the highest performance found among other methods. Of particular note, other methods do not achieve AUC values above 0.8 in A classes, whereas the proposed method showed outstanding performance with AUC of 0.803 in this class. The overall result of the proposed method was 0.794, and the curve is plotted in Figure 6.

To verify the robustness of the proposed method, the registration performance was additionally evaluated on two databases. One involves image datasets with pairs of different image quality, and the other includes image pairs obtained with different modalities. These databases were applied to check whether the proposed method would perform well on poor quality and multimodal images. As shown in Figure 6, the proposed method showed a significant AUC of 0.821 on the different image quality database. High performance was also demonstrated with the multimodal images, with 0.824 and 0.819 for normal and abnormal, respectively.

## 5. Discussion and Conclusion

This study presents a robust detection model of vascular landmarks for retinal image registration. This model involved two convolutional neural networks which were named VSN and JDN. The former segmented retinal vessel on the retinal image, and the latter was used for detecting junction points from the vessel image. Especially, JDN was designed to output the specific areas which include the junction points, and it was calibrated by taking into account that three or more branches are meet in vascular junction points to improve the detection performance. The detected vascular landmarks were applied for image registration to find the same points in image pairs and match them. The proposed method was evaluated using different databases and evaluation metrics for vessel segmentation, junction detection, and registration. This study applied a total of five public databases and seven types of evaluation metrics for quantitative and comparative analysis.

The proposed vascular landmark detection model showed superior results for retinal vessel segmentation and junction detection. First, the proposed VSN segmented the retinal vessel region with better performance compared to other unsupervised/supervised methods with the highest accuracy and AUC which estimate overall performance. The sensitivity of the VSN was 0.805, and this indicates that the proposed network segmented the vessel regions well. Achieving a specificity of 0.982 meant that most nonvessel pixels were predicted as actual class. The JDN, which is the second part of the proposed model, also showed remarkable performance in detecting junction points. It acquired the highest results when using the vessel image as the input image among the three types of the images. This experimental result seems to indicate that the vessel image involves more distinct vessel information than RGB and grayscale images.

The proposed vascular landmark detection model was compared with other state-of-the-art methods on the RetinaCheck database which provides junction information for the DRIVE and IOSTAR image datasets. Although the proposed model achieved significantly good performance, it showed relatively low precision compared to some methods on the IOSTAR dataset. This is likely to be caused by the ground truth of the database. Whereas this dataset did not check junction points within the optic disc area, the proposed model detected the points in this area. This may have effects on the TP and FP, and it may result in the low precision. Nevertheless, the proposed model showed the highest F1 score on the DRIVE and IOSTAR images compared with other methods.

This study registered retinal image pairs based on the detected junction points. The proposed method acquired outstanding performance on the FIRE database. Of particular note, the significantly superior results were confirmed on the A class. This class has anatomical changes between images; thus, this class was registered with low results of under 0.7 in previous studies. In contrast, the proposed method precisely matched the pairs of images by accurately detecting the common points. Therefore, it demonstrated a high performance, and the overall AUC was 0.794 for the FIRE database. However, the proposed method showed relatively low AUC compared with REMPE [53] for the P class. The results may occur because the P class showed low overlap between images. The proposed registered the images with vascular junction points, and the number of these points were relatively small than the keypoints applied in other previous study. Therefore, this limitation may affect the registration performance of P class. Nevertheless, the proposed method showed high performance overall.

Furthermore, this study evaluated the proposed method under various suboptimal image conditions. The proposed method accurately registered poor quality images that were acquired in defocused camera setting with AUC of 0.821. As well, it performed well with images acquired by different modality including fluorescein angiography and retinal image. The AUC values for the multimodal dataset were 0.824 for normal and 0.819 for abnormal. These experimental results verified the clinical effectiveness and robustness of the proposed method for registration of retinal images.

However, this study had limit of the number of dataset. To overcome this limitation, this study tried to acquire as much data as possible by obtaining not only image datasets which have been generally used for fundus image research but also image datasets which have not been applied to related studies. Also, this study organized ground truth datasets by additional labeling task. Although this efforts, it is considered that the limit of the number of data still exists. Therefore, this study will supplement the image dataset with a process of Institutional Review Boards (IRB) in future study, and the proposed method will be evaluated on this rich dataset.

## Figures and Tables

**Figure 1:** The architecture of the vessel segmentation network.

**Figure 2:** The architecture of the multi-input module.

**Figure 3:** The architecture of the connected convolution module.

**Figure 4:** The architecture of the junction detection network. The numbers written after C, M, and P represent the level.

**Figure 5:** The registration results for the retinal images of the S (a–f), P (g–l), and A (m–r) classes on the FIRE database. The first and second columns are original retinal images, and the third to fourth columns are the results of the retinal vessel segmentation and junction detection. The fifth column shows the registration image which marks the area where two images meet as yellow. The last column shows registration result by overlapping images.

**Figure 6:** The error threshold-success rate curve for registration. (a) FIRE database, (b) different quality database from Köhler et al. [32], and (c) multimodal image database from Alipour et al. [33].

**Table 1:** Confusion matrix.

		Predicted class	
		Positive	Negative
Actual class	Positive	TP	FN
	Negative	FP	TN

**Table 2:** Comparison of the segmentation performance on DRIVE database.

Method	Sensitivity	Specificity	Accuracy	AUC
Unsupervised method				
Aguirre-Ramos et al. [34]	0.785	0.966	0.953	—
Shah et al. [35]	0.742	0.977	0.947	—
Memari et al. [36]	0.761	0.981	0.961	0.871
Solís-Pérez et al. [37]	0.827	0.965	0.956	—
Zhou et al. [38]	0.726	0.980	0.948	—
Supervised method				
Zhuang [39]	0.786	0.981	0.956	0.979
Alom et al. [40]	0.779	0.981	0.956	0.978
Guo et al. [41]	0.789	0.980	0.956	0.981
Feng et al. [42]	0.762	0.981	0.953	0.968
Kushol et al. [43]	0.759	0.975	0.946	—
Adapa et al. [44]	0.629	0.984	0.945	0.951
Jin et al. [45]	0.739	0.983	—	0.976
Khan et al. [46]	0.825	0.979	0.965	0.978
Proposed method	0.805	0.982	0.966	0.982

**Table 3:** Detection results of JDN on RetinaCheck database.

Input image type	Precision	Recall	F1 score
Color image	0.723	0.784	0.752
Grayscale image	0.750	0.800	0.774
Vessel image	0.809	0.853	0.831

**Table 4:** Comparison of the detection performance on RetinaCheck database.

Method	DRIVE			IOSTAR		
	Precision	Recall	F1 score	Precision	Recall	F1 score
Azzopardi and Petkov [47]	0.400	0.740	0.520	0.630	0.330	0.430
Abbasi-Sureshjani et al. [30]	0.750	0.610	0.670	0.470	0.600	0.520
Uslu and Bharath [48]	0.650	0.690	0.670	0.520	0.670	0.590
Zhao et al. [49]	0.710	0.700	0.700	0.620	0.570	0.600
Proposed method	0.805	0.776	0.790	0.524	0.842	0.646

**Table 5:** Comparison of the fundus image registration performance on FIRE database.

Method	Classes of FIRE data		
	S	P	A
SIFT [13]	0.967	0.411	0.534
SURF [50]	0.978	0.384	0.422
GDB-ICP [51]	0.814	0.303	0.303
Harris-PIIFD [3]	0.900	0.090	0.443
H-M 16 [52]	0.945	0.443	0.577
REMPE [53]	0.958	0.542	0.660
Proposed method	0.988	0.511	0.803

## Data Availability

The datasets that were used in this study are openly available in the DRIVE database (http://www.isi.uu.nl/Research/Databases/DRIVE/) [28], RetinaCheck database (http://www.retinacheck.org/) [29, 30], IOSTAR database [29, 30], FIRE database (https://projects.ics.forth.gr/cvrl/fire/) [31], HRF database (https://www5.cs.fau.de/research/data/fundus-images/) [32], and Fundus Fluorescein Angiogram Photographs and Colour Fundus Images of Diabetic Patients database (https://hrabbani.site123.me/available-datasets/) [33].
